# Proteomic Analysis of Lung Tissue in a Rat Acute Lung Injury Model: Identification of PRDX1 as a Promoter of Inflammation

**DOI:** 10.1155/2014/469358

**Published:** 2014-06-15

**Authors:** Dongdong Liu, Pu Mao, Yongbo Huang, Yiting Liu, Xiaoqing Liu, Xiaoqing Pang, Yimin Li

**Affiliations:** ^1^State Key Laboratory of Respiratory Diseases, The First Affiliated Hospital of Guangzhou Medical University, 151 Yanjiang West Road, Guangzhou, Guangdong 510120, China; ^2^Intensive Care Unit, The First Affiliated Hospital of Guangzhou Medical University, Guangzhou, China; ^3^Infection Control Department, The First Affiliated Hospital of Guangzhou Medical University, Guangzhou, China

## Abstract

Acute respiratory distress syndrome (ARDS) remains a high morbidity and mortality disease entity in critically ill patients, despite decades of numerous investigations into its pathogenesis. To obtain global protein expression changes in acute lung injury (ALI) lung tissues, we employed a high-throughput proteomics method to identify key components which may be involved in the pathogenesis of ALI. In the present study, we analyzed lung tissue proteomes of *Pseudomonas aeruginosa*-induced ALI rats and identified eighteen proteins whose expression levels changed more than twofold as compared to normal controls. In particular, we found that PRDX1 expression in culture medium was elevated by a lipopolysaccharide (LPS) challenge in airway epithelial cells *in vitro*. Furthermore, overexpression of PRDX1 increased the expression of proinflammatory cytokines interleukin-6 (IL-6), interleukin-8 (IL-8), and tumor necrosis factor-*α* (TNF-*α*), whereas knockdown of PRDX1 led to downregulated expression of cytokines induced by LPS. In conclusion, our findings provide a global alteration in the proteome of lung tissues in the ALI rat model and indicate that PRDX1 may play a critical role in the pathogenesis of ARDS by promoting inflammation and represent a novel strategy for the development of new therapies against ALI.

## 1. Introduction

Acute lung injury (ALI) and its more severe form, acute respiratory distress syndrome (ARDS), are the major causes of death in critically ill patients. Despite significant improvements in diagnosis and supportive care, the mortality of ARDS remains as high as approximately 40% [1]. Evidently, a better understanding of the molecular mechanism underlying ARDS from an overall perspective is needed.

The pathophysiologic course of ARDS is characterized by overwhelming lung inflammation, inappropriate accumulation and activity of leukocytes and platelets, uncontrolled activation of coagulation pathways, and increased permeability of alveolar endothelial and epithelial barriers [2]. ARDS is a complex clinical disorder developed from a variety of severe conditions such as sepsis, severe pneumonia, and trauma [3]. It is believed that a number of genes are involved in the development of ARDS [4], thereby forming a complete signaling pathway network. Signal pathways regulating innate immunity and antibacterial defenses play a critical role in the development of ARDS [5, 6]. Other pathways regulating angiotensin-converting enzyme 2 and lipid modifications are also implicated in the pathogenesis of ARDS [7–9]. Although numerous studies investigating the pathogenesis of ARDS have been published during the last decades, most of them mainly addressed a single perspective involved in ARDS and could not offer an overall view. Thus there remain significant challenges in elucidating the molecular mechanisms underlying ARDS.

In order to obtain an overview of the molecular pathogenesis of ARDS, high-throughput assays, including mRNA profiles, metabolomics, genetic studies, and proteomics, are required. Proteomics is a high-throughput method that can compare the overall proteins of cells and tissues under different conditions to identify deregulated proteins which may be key mediators of pathogenesis or biomarkers of disease progress or outcome [10, 11]. Studies on proteomics in ALI/ARDS have been reported [12]. For example, Ménoret A et al. identified cytochrome b5 and cytokeratin 17 as early markers of ALI in a rats model by using the proteomic PF 2D platform [13]; Schnapp et al. analyzed bronchoalveolar lavage fluid (BALF) from three ALI patients by using proteomics and found that the insulin-like growth factor-binding protein-3 (IGFBP-3) concentration was increased in the BALF from ALI patients when compared to normal controls [14]. By analyzing the changes in protein expression in the BALF of ARDS patients, Chang et al. identified 22 proteins whose expressions had changed and were significantly increased in processes involved in inflammation, immunity, responses to microbials and stress, and/or injury [15]. However, most of comparative proteomic studies reported previously on the pathogenesis of ALI/ARDS were mainly focused on the protein alterations in BALF. As far as we know, no studies on proteomic changes in ALI lung tissue have been reported.

The present study employed a rat model of* Pseudomonas*-induced acute lung injury and utilized a comparative proteomics approach to identifying differentially expressed proteins in the lung tissue in the course of ALI. Protein alterations were identified by MALDI-TOF-MS, and the mRNA and protein expression levels of peroxiredoxin1 (PRDX1) whose expression was markedly increased in the ALI rat lungs were further confirmed by real-time PCR and western blotting analysis. The upregulation of PRDX1 and its biological function were also elucidated in a LPS-induced airway epithelium cell injury model* in vitro*.

## 2. Materials and Methods

### 2.1. Cell Line

The BEAS-2B immortalized human bronchial epithelial cell line was purchased for the American Type Culture Collections (ATCC, Rockville, MD). Cells were cultured as previously described [16], maintained in 75 cm^2^ flasks in DMEM/F-12 (Invitrogen, Carlsbad, CA), and supplemented with 10% fetal bovine serum (FBS) (HyClone, Logan, UT), in a 95% humidified air incubator, set at 37°C, with 5% CO_2_.

### 2.2. Antibody and Reagent

Oleic acid and lipopolysaccharides (LPS,* Pseudomonas aeruginosa* 10) were purchased from Sigma-Aldrich (St. Louis, MO). Rabbit polyclonal anti-peroxiredoxin 1 antibody was purchased from Abcam (Cambridge, MA). Antibody for NF-*κ*B p65 and *β*-actin was purchased from Santa Cruz Biotechnology (Santa Cruz, CA). Antibody for *α*-tubulin was purchased from Sigma-Aldrich (St Louis, MO).

### 2.3. Animal Models

All animal protocols were approved by the Experimental Animal Ethics Committee of the Guangzhou Medical University. Sixty adult specific pathogen-free male Sprague Dawley rats (250–300 g) were obtained from the Medical Laboratory Animal Centre of Guangdong Province (Guangzhou, China). The rats were housed in individual cages in a temperature-controlled room with alternating 12 h light/dark cycles and acclimated for one week before the study. Food was removed eight hours prior to the study, but all animals had free access to water. All animals were anesthetized with pentobarbital (50 mg/kg, intraperitoneal injection). The rats were randomly separated into two groups: control group (*n* = 15) and a* Pseudomonas* group (*n* = 15). The* Pseudomonas*-induced acute lung injury rat model was generated according to the methods reported previously [17, 18]. Briefly, the* Pseudomonas* rat model was induced via intratracheal injection of 0.3 mL phosphate-buffered saline (PBS) containing* Pseudomonas* (9 × 10^8^ colonies forming units/mL). The animals were killed by exsanguination under anesthesia 24 h later.

### 2.4. Assessment of Acute Lung Injury

Lung tissues from eight animals in each group were taken for histopathology. The lungs were fixed in 4% paraformaldehyde, embedded in paraffin, sectioned, and stained with haematoxylin-eosin (HE) according to standard methods. The lung injury was assessed with a modified scoring system according to alveolar collapse, alveolar hemorrhage, perivascular edema, alveolar edema, polymorphonuclear leukocyte infiltration, and cellular exudates in a blinded fashion [19]. Scoring categories were none, mild, moderate, and severe (scores 0, 1, 2, and 3, resp.). The mean score for each pathologic parameter was calculated.

### 2.5. Preparation of BALF and Measurements

After animals were sacrificed, tracheotomy was conducted (seven rats per group), and a 22-gauge catheter was inserted into the trachea. With the right bronchus ligated, the left lung was lavaged with 2 mL of 4°C PBS three times. The recovered lavage fluids were centrifuged for 10 min at 5,000 rpm and the supernatants were stored at −80°C until further analysis. The BALF was diluted two times for concentration measurements. Concentrations of TNF-*α* and interleukin-1*β* (IL-1*β*) in the BALF supernatants were measured using rat-specific ELISA kits (R&D Systems, Minneapolis, MN) in accordance with the manufacturer's instructions.

Wet-to-dry weight ratios (W/D) were measured as described previously [20]. In short, after the experiment the lungs were excised en bloc. The tissue sample weights were obtained immediately to prevent evaporative fluid loss from the tissues. Lungs were then dried in an oven at 80°C for 72 h and the dry weight was measured. W/D ratios were then calculated as milligrams of water per milligram of dry tissue.

### 2.6. Protein Preparation

Lung tissues were washed twice with cold PBS. Lung tissue was ground into powder in liquid nitrogen. The powder was then put into a prechilled EP tube and homogenized after adding lysis buffer containing 0.5 mM ethylenediaminetetraacetic acid (EDTA), 7 M urea, 2 M thiourea, 4% CHAPS detergent, 2 mM dithiothreitol (DTT), and 2 mM phenylmethanesulfonyl fluoride (PMSF). After standing at room temperature for 30 min, the homogenate was centrifuged at 17000 g/min at 4°C for 90 min. The supernatant containing the tissue protein was then collected, and the concentration of proteins was measured using a Bradford protein quantification kit (Bio-Rad Protein Assay, Bio-Rad, Richmond, CA).

### 2.7. IEF and Electrophoresis

The lung homogenate (850 *μ*g of protein) was mixed with rehydration buffer (7 M urea, 2 M thiourea, 4% CHAPS, 2 mM DTT, and 2% immobilized pH gradient (IPG) buffer). Protein samples were directly applied to IPG strips (pH 3–10, 17 cm) and rehydrated for 12 h at room temperature. Next, isoelectric focusing (IEF) was performed using the IPGphor (Bio-Rad, Richmond, CA) apparatus. IEF was performed for a total of 80 kVh (the initial voltage was maintained at 150 V for 1 h, 250 V for 1 h, linearly increased from 500 to 5000 V within 3.5 h, ramped to 10 000 V in 5 h, and maintained at 10 000 V for 60 kVh). The IPG strips were incubated in equilibration buffer (6 M urea, 2% sodium dodecyl sulfate (SDS), 1.5 M pH = 8.8 Tris-Cl, 20% glycerol) supplemented with 0.5% DTT for 15 min at room temperature and followed by a 15 min incubation in equilibration buffer with 2.5% iodoacetamide at room temperature. Equilibrated strips were directly loaded onto 12% polyacrylamide gels; then the second dimension SDS-PAGE (polyacrylamide gel electrophoresis) was carried out at 20 mA per gel with the Protean II xi Cell system (Bio-Rad, Richmond, CA).

### 2.8. Staining and Image Analysis

After SDS-PAGE, gels were fixed and protein spots were visualized by Coomassie brilliant blue staining. The 2-DE images were scanned by Image Scanner II and analysed with Image Master 2D Elite 5.0 software (Amersham Biosciences, Buckinghamshire, UK). To confirm the variations, at least three gels were prepared for every case. Computer analysis facilitated the automatic detection and quantification of protein spots, as well as matches between gels of control groups and* Pseudomonas* groups. Spots displaying reliable and significant differences (± over twofold, *P* < 0.05) were selected for MS analysis.

### 2.9. In-Gel Digestion

Coomassie blue-stained protein spots on the polyacrylamide gel were excised and transferred into a 0.5 mL microcentrifuge tube, rinsed twice with ddH_2_O, and then destained in a 1 : 1 solution of 100 mM ammonium bicarbonate and acetonitrile. After hydrating with acetonitrile and drying in a SpeedVac centrifuge, the gels were rehydrated in a minimal volume of sequencing grade porcine trypsin (Promega, Madison, WI) solution (20 *μ*g/mL in 25 mM NH_4_HCO_3_) and incubated at 37°C overnight. The supernatants were transferred into a 200 *μ*L microcentrifuge tube and the gels were extracted once with extraction buffer (67% acetonitrile containing 1% trifluoroacetic acid). The peptide extract and the supernatant of the gel spot were combined and then completely dried in a SpeedVac centrifuge.

### 2.10. MALDI-TOF/TOF Analysis and Database Searching

Protein digestion extracts (tryptic peptides) were resuspended with 5 *μ*L of 0.1% trifluoroacetic acid and the peptide samples were mixed (1 : 1 ratio) with a matrix consisting of a saturated solution of *α*-cyano-4-hydroxy-trans-cinnamic acid in 50% acetonitrile-1% trifluoroacetic acid. Aliquots of 0.8 *μ*L were spotted onto stainless steel sample target plates. Peptide mass spectra were obtained from an Applied Biosystem Sciex 4800 MALDI TOF/TOF mass spectrometer. Data were acquired in a positive MS reflector using a Cal Mix 5 standard to calibrate the instrument (ABI4700 Calibration Mixture). Mass spectra were obtained from each sample spot by accumulation of 600–800 laser shots in an 800–4000 mass range. For MS/MS spectra, the five most abundant precursor ions per sample were selected for subsequent fragmentation and 900–1200 laser shots were accumulated per precursor ion. The criterion for precursor selection was a minimum signal-to-noise ratio (S/N) of 50. Both the MS and MS/MS data were interpreted and processed by using the GPS Explorer software (V3.6, Applied Biosystems). The obtained MS and MS/MS spectra per spot were combined and submitted to the MASCOT search engine (V2.1, Matrix Science, London, UK) by GPS Explorer software and searched with the following parameters: Database—Rat International Protein Index (IPI) v3.52; Digestion Enzyme—trypsin; Missed cleavage site—one; Partial modification—cysteine carboamidomethylated and methionine oxidized; Fixed modifications—none selected; MS tolerance—50 ppm; MS/MM tolerance—0.25 Da. Known contaminant ions (keratin) were excluded. A total of 69012 sequences and 29002682 residues in the database were actually searched. MASCOT protein scores (based on combined MS and MS/MS spectra) of greater than 61 were considered statistically significant (*P* ≤ 0.05). The individual MS/MS spectra with statistically significant (confidence interval >95%) best ion score (based on MS/MS spectra) were also accepted.

### 2.11. Western Blotting Analysis

Western blotting was used to verify differentially expressed proteins. Proteins were separated by 12% SDS-PAGE gel and transferred onto polyvinylidene difluoride (PVDF) membranes at 300 mA for 90 min. Membranes were blocked with 5% nonfat milk in TBST buffer for 1 h at room temperature with gentle rocking and then probed with antibodies. Membranes were incubated with the primary antibody at 4°C overnight with gentle rocking. The membranes were then washed three times with tris-buffered saline and Tween 20 (TBST buffer) for 15 min and incubated with horseradish peroxidase (HRP) conjugated secondary (dilution, 1 : 20000) for 1 h at room temperature. The hybridized membrane was washed in TBST buffer, visualized using an enhanced chemiluminescent (ECL) detection kit (Abcam, Cambridge, MA), and exposed to X-ray film.

To detect PRDX1 in culture medium of BEAS-2B cells by western blotting, cells grown in 60 mm dishes were washed three times with serum-free DMEM/F-12 and then covered with 3 mL of 1% FBS DMEM/F-12 with or without LPS. The conditioned media were collected and centrifuged at 1500 rpm for 5 min for removal of nonadherent cells and debris. The supernatants were concentrated to a final volume of 50 *μ*L. The concentrated culture media were used to detect the presence of PRDX1 by western blotting analysis.

### 2.12. Immunohistochemistry Analysis (IHC)

The IHC procedure was carried out as previously reported [21]. In brief, paraffin-embedded specimens were cut into 4 *μ*m sections and baked at 65°C for 30 min. Sections were deparaffinized with xylene and rehydrated. Sections were submerged into EDTA antigenic retrieval buffer and microwaved for antigenic retrieval. The sections were treated with 3% hydrogen peroxide in methanol to quench the endogenous peroxidase activity, followed by incubation with 1% bovine serum albumin to block nonspecific binding. Rabbit anti-peroxiredoxin 1 (1 : 800, Abcam, Cambridge, MA) was incubated with the sections overnight at 4°C. After washing, the tissue sections were treated with biotinylated anti-rabbit secondary antibody (Zymed, South San Francisco, CA), followed by further incubation with streptavidin-horseradish peroxidase complex (Zymed, South San Francisco, CA). The tissue sections were immersed in 3-amino-9-ethyl carbazole and counterstained with hematoxylin. The specificity of antibodies was determined by replacing the primary antibody with nonimmunized IgG.

### 2.13. Reverse Transcriptase-Polymerase Chain (RT-PCR) Reaction Assay

Trizol reagent (Invitrogen, Carlsbad, CA) was added to samples for extraction of total RNA. The PrimeScript RT-PCR kit (Takara Bio Company, Shanghai, China) was employed to synthesize cDNA, and expression of peroxiredoxin 1. The proinflammatory cytokines IL-6, IL-8, and TNF-*α* mRNA were examined through polymerase chain reaction (PCR). Primers used to amplify the conserved regions of the genes of interest in BEAS-2B cells are shown in Table 1. PCR products were resolved into a 1% agarose gel, stained with ethidium bromide, and photographed under ultraviolet illumination. The band intensity was quantified by Quantity One Software (Bio-Rad, Richmond, CA).

### 2.14. Enzyme-Linked Immunosorbent Assay (ELISA) for PRDX1

The conditioned medium was collected and centrifuged at 1500 rpm for 5 min to remove cell debris. PRDX1 concentration was measured using PRDX1 (Human) ELISA Kit (Abnova, Taiwan) according to the manufacturer's instructions. The conditioned medium was diluted 1 : 2 prior to measurement and was assayed simultaneously and in duplicate. Serial dilutions of PRDX1 standard were assayed in parallel with medium samples. The optical density was plotted against standard PRDX1 concentrations to generate the standard curve according to the manufacturer's protocol.

### 2.15. Cell Viability Assay

Cell viability was evaluated by MTT assay as previously described [22]. To evaluate the effect of LPS on cell viability, BEAS-2B cells were seeded in 96-well plates at 5 × 10^4^ cells/well for 24 h. The cells were treated with the two concentrations of LPS (1 and 10 *μ*g/mL) for 12 h and 24 h at 37°C, respectively. At the end of exposure, 40 *μ*L of MTT solution (2 mg/mL) was added and the cells were incubated for 4 h at 37°C. Cells were treated with 150 *μ*L of dimethylsulfoxide (DMSO) and absorbance was quantified at 540 nm. The viability of the treated group was expressed as a percentage of nontreated control group, which was assumed to be 100%.

### 2.16. Plasmids and Transfection

The PRDX1 construct was generated by subcloning PCR-amplified full-length human PRDX1 cDNA into the vector plasmid pMSCV. For depletion of PRDX1, 5 human siRNA sequences were cloned into the pSuper retro puro plasmid to generate pSuper retro PRDX1-RNAi(s), and the sequences were RNAi#1: CAGCCTGTCTGACTACAAAGG; RNAi#2: GCACCATTGCTCAGGATTATG; RNAi#3: AGGGTATTCTTCGGCAGATCA; RNAi#4: GCTCTGTGGATGAGACTTTGA; RNAi#5: GTTCTCCGAACGTGTCACGTC. Transfection of plasmids was carried out by using the Lipofectamine 2000 Reagent (Invitrogen, Carlsbad, CA) according to the manufacturer's instruction.

### 2.17. Statistical Analysis

Data are presented as mean ± SD. Analysis of variance was used to evaluate differences between the groups. Experimental data for 2-DE were analyzed using Image Master 2D Elite 5.0 Software and Student's *t*-test. *P* value less than 0.05 was considered statistically significant.

## 3. Results

### 3.1. Evaluation of Lung Injury

Morphological changes in lung tissues were examined to determine whether the acute lung injury rat models were established. HE staining showed that no sign of lung damage was observed in the control group, as shown in Figure 1(a). However, the* Pseudomonas* group showed hemorrhage and interstitial edema after 24 hours, and infiltrations of inflammatory cells were observed in most of the alveolar spaces. In conjunction with histological changes of the lung tissues, the lung injury score was also significantly higher in the lung injury group, as compared to the control group (Figure 1(b)).

To further evaluate the lung injury, pulmonary W/D data and levels of TNF-*α* and IL-1*β* in the BALF were assessed. These reflect the pulmonary edema severity and inflammation level, respectively. Consistent with histological changes and lung injury score, pulmonary W/D data and the levels of TNF-*α* and IL-1*β* in BALF in the injury group were much higher than those in the control group (*P* < 0.05), as shown in Figures 1(c), 1(d), and 1(e), respectively. These findings demonstrated that the current model is suitable to be used to investigate the differentially expressed proteins of ALI.

### 3.2. Proteomic Analysis of Lung Tissue of ALI Rat Model

To investigate the molecular mechanism of* Pseudomonas*-induced lung injury, we performed a quantitative proteomic approach to evaluating changes in lung tissue proteomes. After 2-DE, the gels were scanned and analyzed with Image Master 2D Elite 5.0 software. An average of 900 protein spots was found on each gel according to the results of the image analysis. Among the 878 matched protein spots, 25 protein spots in the* Pseudomonas* group showed greater than twofold differences (all *P* < 0.05) as compared to the control. These protein spots were picked up and were then subjected to in-gel digestion and further analyzed with MALDI-TOF-MS. Eighteen proteins differentially expressed between the lung injury and control group were identified (Table 2 and Figure 2). Eleven proteins were upregulated and 7 proteins were downregulated in the* Pseudomonas* ALI groups. The proteins are involved in various biological processes according to gene ontology, including metabolic processes (33.3%, 6/18), protein binding (38.9%, 7/18), signal transduction (11.1%, 2/18), and antioxidant activity (16.7%, 3/18). Peroxiredoxin 1 (PRDX1), calreticulin, superoxide dismutase 2, nucleoside diphosphate kinase B, and aldolase A were overexpressed in the* Pseudomonas* groups, whereas apolipoprotein E, glutathione S-transferase alpha 4, and RAKC protein showed lower expression levels.

### 3.3. Validation of PRDX1 Expression by Real-Time PCR, Western Blot, and Immunohistochemistry

PRDX1 is a member of the peroxiredoxin family that is nonclassically secreted from cells and acts as a mediator of inflammation in prostate cancer [23, 24]. Therefore, specific attention was paid to PRDX1 which showed the most robust change in expression (4.79-fold increase; Table 2) in the current study. To verify proteomic results and assess the expression change of PRDX1 showing differential patterns in* Pseudomonas*-induced acute lung injury, real-time PCR, western blot, and immunohistochemistry were performed. As shown in Figure 3, both the protein level and mRNA level of PRDX1 were increased in the* Pseudomonas*-induced lung injury group, which was consistent with results from the proteomic experiments.

### 3.4. LPS Causes Upregulation of PRDX1 in Culture Medium of BEAS-2B Cells

Our previous study found that PRDX1 expression could be elevated under LPS treatment in a human bronchial epithelial cell line BEAS-2B [25]. It is reported that PRDX1 could be secreted from tumor cells and extracellular PRDX1 could induce the secretion of proinflammatory cytokines such as TNF-*α* and IL-6 [26]. Therefore, we examined whether concentration of PRDX1 is upregulated in culture medium in bronchial epithelial cells under the challenge of LPS. We used BEAS-2B cells as a representative airway epithelial cell line to establish the LPS-induced acute lung injury cell model. A dramatic morphological change was observed in the BEAS-2B cells after a challenge with LPS for 24 hours at a concentration at 10 *μ*g/mL (Figure 4(a)). As shown in Figure 4(b), BEAS-2B cell viability was decreased by treatment with LPS in dose-dependent manner at 24 hours. Taken together, these results indicated that the cell injury model was established. Conditioned media were analyzed by western blotting and we observed a significant increment in PRDX1 expression in culture media at 12 and 24 hours after 1 *μ*g/mL and 10 *μ*g/mL of LPS treatment (Figure 4(c)). *α*-Tubulin was not detected in the conditioned media (Figure 4(c)) indicating the absence of cell lysis. We also detected the concentration of PRDX1 in media by ELISA and results demonstrated that the concentration of PRDX was increased in a dose-dependent manner after LPS treatment as compared to the control (Figure 4(d)). These results indicated that the expression level of PRDX1in culture medium was increased under the exposure of LPS in lung epithelium cells.

### 3.5. PRDX1 Expression Modulated Inflammation in Airway Epithelium Cells

In order to explore the significance of PRDX1 upregulation in acute lung injury, a PRDX1 expressing vector and a PRDX1 sequence specific shRNA expression vector were constructed and transduced to the BEAS-2B cell. As shown in Figure 5(a), the protein level of PRDX1 was increased under the pPSCV-PRDX1 transduction as compared to the vector transduction. We next determined the effect of PRDX1 overexpression on IL-6, IL-8, and TNF-*α* after LPS treatment in BEAS-2B cells. PRDX1 overexpressed BEAS-2B cells showed a significant increase of IL-6, IL-8, and TNF-*α* expression compared to the control group. This is similar to the results of LPS treatment on vector transduced BEAS-2B cells. PRDX1 overexpressed cells did not show further increase of IL-6, IL-8, and TNF-*α* expression after challenge with LPS, indicating that PRDX1 expression alone could upregulate the inflammation in BEAS-2B cells.

Furthermore, the impact of PRDX1 expression on cytokine expression was evaluated in PRDX1 knockdown BEAS-2B cells. Four pSUPER-PRDX1 shRNA plasmids were constructed and then transfected into the BEAS-2B cells and results showed that transfection with the shRNA#3 led to the marked reduction of PRDX1 expression (Figure 5(b)). Therefore, shRNA#3 was used in the following experiments. As shown in Figure 5(d), the depletion of PRDX1 expression caused considerable downregulation of IL-6, IL-8, and TNF-*α* expression in PRDX1 shRNA transduced BEAS-2B cells compared to vector transduced cells with LPS treatment. Moreover, treatment with LPS in PRDX1 knockdown BEAS-2B cells did not show an increase of IL-8 and TNF-*α* expression. These results implying PRDX1 might play a role in LPS-induced inflammation in lung airway cells.

The NF-*κ*B signaling pathway is known to play a critical role in the regulation of inflammatory cytokine production. Thus, we investigated whether the PRDX1 expression altered the nuclear translocation of NF-*κ*B. Nucleic fractions of the cell lysates were extracted and the expression of p65 protein was analyzed by western blotting analysis. As shown in Figure 5(e), expression of PRDX1 increased the amount of NF-*κ*B p65 protein in the nuclear fraction, whereas knockdown of PRDX1 by shRNA reduced nucleus accumulation of the p65 protein. This suggests that PRDX1 expression modulated the expression of cytokines through the NF-*κ*B signaling pathway.

## 4. Discussion

In the current study, we employed a high-throughput proteomic approach to identifying the global proteome alterations of lung tissue using a rat model with bacterially induced acute lung injury. Proteomic analysis revealed 18 differentially expressed proteins, of which 11 were upregulated and 7 were downregulated in ALI lung tissues, as compared to the normal control. These differentially expressed proteins were mainly associated with cellular metabolism, antioxidation, signal transduction, and protein binding. PRDX1 overexpression was verified by western blot, real-time PCR, and IHC analysis. An* in vitro* study using an airway epithelium cell model showed that PRDX1 expression was upregulated in culture medium under the challenge of LPS. Moreover, overexpression of PRDX1 and knockdown of its expression promoted and inhibited the production of proinflammatory cytokines, respectively. Finally, our results indicated that PRDX1 promoted inflammatory processes via the NF-*κ*B signaling pathway. Findings from the current study provide a novel insight into the mechanisms underlying bacterially induced ALI.

It has been reported that diffuse increase in metabolic activity is observed in the lungs of ALI and ARDS patients and that this increased activity indicates the presence of an inflammatory process [27, 28]. In the current study, changes in eight proteins that were involved in cellular metabolism were identified, as shown in Table 2. These results strongly suggest that significant metabolic dysregulation occurs in* Pseudomonas*-induced acute lung injury, perhaps because of the existence of inflammation and excessive epithelium and endothelium damage in lungs of ALI patients. Among other differentially expressed proteins, several proteins have been reported to be involved in the pathogenesis of ALI. For example, Rho-associated protein kinase 1 (ROCK), which is the downstream target of Rho GTPases, is believed to play an important role in the regulation of the endothelial cell actin cytoskeleton. It is a mediator of TNF-*α* and vascular endothelial growth factor- (VEGF-) induced endothelial hyperpermeability and vascular barrier dysfunction, which are both key ALI pathophysiological characteristics [29, 30]. Calreticulin (CRT), a multifunctional endoplasmic reticulum luminal Ca^2+^-binding chaperone, was found to stimulate the antioxidant pathway and was able to protect A549 human type II alveolar epithelial cells by diminishing reactive oxygen species (ROS), which are key signaling molecules mediating many types of cell injury [31, 32]. Furthermore, CRT gene expression was significantly upregulated in catfish under the challenge of infectious gram-negative bacteria through reducing excess ROS [33]. A study shows that the concentration of hemoglobin in the BALF was significantly increased in ARDS patients [34]. However, whether the rest of the proteins which showed differential expression play roles in the pathogenesis of ALI or just act as innocent bystanders remains unknown and needs further investigation.

Peroxiredoxin 1 (PRDX1), a finding worthy of note, was the top overexpressed protein in the bacterially infected group relative to the control group, thus encouraging us to explore what specific role PRDX1 may be involved with in the development of ARDS. Therefore, we validated the overexpression of PRDX1 by RT-PCR, western blot, and immunohistochemistry in the lung tissue from ALI rats. We also found that the overexpression of PRDX1 was mainly observed in airway epithelial cells, which are the primary defensive barrier against various attacks from the external environment and thus are frequently injured in ARDS. Our previous study demonstrated that PRDX1 expression was elevated under LPS treatment in a human bronchial epithelial cell line BEAS-2B. Here, we further studied whether the expression of PRDX in the culture medium could be increased under the challenge of LPS* in vitro*. Our results demonstrated that PRDX1 expression in culture medium was substantially upregulated under the challenge of LPS. Interestingly, although the treatment with LPS at 12 hours did not cause significant cell death in BEAS-2B cell, the expression level of PRDX1 in conditioned media after LPS treatment at 12 hours was even higher than that in conditioned media after LPS treatment at 24 hours. Thus, we speculate that extracellular PRDX1 in culture medium is mainly secreted from live cells rather than released from dead cells. It is reported that various oxidative stress stimuli including hydrogen peroxide and sulfhydryl reactive agents are able to upregulate the PRDX1 gene expression in mouse peritoneal macrophages [35, 36]. Treatment of LPS in epithelial cells or macrophages results in production of reactive oxygen species (ROS) which causes oxidative stress [37, 38] and Nrf1 (NF-E2 related factor-1) and Nrf2 (NF-E2 related factor-2), two oxidative stress-sensitive transcription factors, interact with MafG to upregulate the transcription of many antioxidant genes including PRDX1 when activated by oxidative stress [39–41]. Therefore, upregulation of PRDXI gene expression by LPS in BEAS-2B cells is considered to be a cellular response to oxidative stress. Another study also indicated the upregulation of PRDX1 by LPS treatment involved with the Src/PI3 K/JNK signaling pathway which was activated by the treatment of LPS in RAW 264.7 cells [26].

We then modulated the expression of PRDX1 in BEAS-2B cells in order to study the effects of PRDX1 expression on the ability to influence LPS-induced inflammatory processes in the airway epithelium. Surprisingly, results showed that overexpression of PRDX1 in BEAS-2B cells significantly leads to increases in levels of the proinflammatory cytokines IL-6, IL-8, and TNF-*α*, and knockdown of PRDX1 expression inhibited the expression of these cytokines, even under the challenge of LPS. Overall, our results revealed that high expression of PRDX1 might be an important mediator of LPS-induced lung epithelial cell injury.

PRDX1 is a member of the typical 2-cysteine peroxiredoxin family, whose major intracellular functions are as a protein chaperone and a regulator of hydrogen peroxide signaling through its peroxidase activity [42]. Peroxiredoxins efficiently catalyze the breakdown of H_2_O_2_ and alkyl peroxides to eliminate intracellular ROS produced in response to epidermal growth factor and tumor necrosis factor alpha stimulation [43]. However, besides its intracellular functions as a member of the peroxidase family and a protein chaperone [44], PRDX1 can be secreted via a nonclassical secretory pathway by non-small cell lung cancer cells [24, 35]. It has been showed that extracellular PRDX1 acted as a toll-like receptor 4 (TLR4) ligand and stimulated secretion of proinflammatory cytokines TNF-*α* and IL-6 from macrophages and dendritic cells [36]. Shichita et al. also demonstrated that the peroxiredoxin family, including PRDX1, contributed to the induction of inflammatory cytokines in macrophages and extracellular peroxiredoxins are danger signals in the ischemic brain [37]. This suggests that PRDX1 may function as an endogenous damage-associated molecular pattern molecule (DAMP). Interestingly, the PRDX1 level in the BALF of ARDS patients was much higher as compared to healthy controls [38]. Taken together, we propose that PRDX1 expression level is upregulated in airway epithelial cells which are extensively damaged in ALI by various insults, such as LPS, and it is subsequently secreted from the epithelium to act as a DAMP to promote inflammation in the process of ALI.

Finally, previous investigation has reported that extracellular PRDX1 could motivate the TLR-MyD88 signaling pathway by binding to TLR4, which leads to nuclear translocation and activation of the NF-*κ*B pathway [26]. We showed that overexpression of PRDX1 promotes nuclear translocation of p65, and conversely knockdown of PRDX1 expression by shRNA in BEAS-2B cells results in reduction of p65 expression in the nucleus. Thus, our results provide evidence in support of the hypothesis that PRXD1 increases the expression of proinflammatory cytokines by activating the NF-*κ*B pathway. PRDX1 plays multifaceted roles in regulating NF-*κ*B signaling pathway dependent on its subcellular compartments. It is a well-known fact that cytosolic PRDX1 scavenges the ROS such as intracellular H_2_O_2_ to block the activation of NF-*κ*B signaling pathway [39, 40]. However, the functions of PRDX1 are not restricted to its antioxidant activity. Secretory PRDX1 functions in extracellular space independent of its peroxidase activity. Extracellular PRDX1 binds to the surface TLR4 resulting in activation of NF-*κ*B and acts as a proinflammatory factor [26, 41]. Thus, therapies targeting extracellular PRDX1, such as utilization of neutralizing antibody against PRDX1, might be an effective way to attenuate the inflammation response in ALI.

We acknowledge that the present study has some limitations. First, we did not use PRDX1-deficient animals to strongly demonstrate that PRDX1 contributes to the pathogenesis of* Pseudomonas aeruginosa*-induced ALI. However, a study from other investigators has indicated that PRDX1 null mice exhibited reduced acute lung inflammation in O_3_-induced pulmonary inflammation and suggested that PRDX1 plays a positive role in the development of lung inflammation instead of being an effective protector against O_3_-induced oxidative damages [45]. Second, we did not study the effects of upregulated extracellular PRDX on other cell types such as neutrophil cells and macrophages which also play key roles in the pathogenesis of bacterially infected ALI.

## 5. Conclusion

In conclusion, for the first time, we established the well-reproducible 2-DE profiles of lung tissue proteins in a* Pseudomonas*-induced ALI rat model and revealed the proteomic profile of the lung tissue. Through this proteomic approach, we identified 18 differentially expressed proteins which are mainly involved with energy metabolism, antioxidation, protein binding, and signaling transduction. Further investigation showed that PRDX1 plays a role in the regulation of proinflammatory cytokine expression. Insights gained from current studies indicate that PRDX1 may present a potentially new therapeutic target against ALI.

## Figures and Tables

**Figure 1:** The establishment of the* P. aeruginosa-* (PA-) induced acute lung injury rat model. (a) Representative hematoxylin-eosin-stained lung tissue from the rats. Rats subjected to* P. aeruginosa* showed evidence of extensive lung injury with hemorrhage, inflammatory cell infiltration, and interstitial and alveolar edema compared with control conditions. Lung injury score (b), the lung W/D ratio (c), BALF TNF-*α*, and IL-1*β* ((d) and (e)) concentration were significantly increased in* P. aeruginosa* ALI rats as compared to control rats. *n* = 8 rats/group. *P < 0.05.

**Figure 2:** Proteomic analysis of lung tissue of ALI rat model. (a) Representative 2-DE gel images of lung tissues from control rats (left) and* P. aeruginosa*-infection induced ALI (right). Arrow indicates the spot of PRDX1. (b) A typical MALDI-MS spectrum of spot gi|16923958 from the 2-DE map. The MS spectrum of the peptide mixture was obtained from a typical in-gel digestion of the 2-DE separated protein.

**Figure 3:** The mRNA and protein level of PRDX1 was determined by western blotting (a), real-time PCR (b), and IHC ((c) and (d)), respectively. (a) Expression of PRDX1 protein in lung tissues of ALI and control rats by western blotting. *β*-Actin was used as a loading control. Data are reported as relative densitometry of the PRDX1 over *β*-actin in bar graphs. There is no statistical significance between Control-2 and Control-1, *P < 0.05 versus Control-1. (b) Real-time PCR analysis of PRDX1 mRNA expression in the ALI and control rats. (c) PRDX1 expression levels were upregulated in ALI rat lung tissue in comparison to the control rat lung tissue as examined by IHC, original magnification, ×200. (d) The average MOD of PRDX1 staining between the ALI and control rat lung tissues was statistically quantified. (b) and (d): *n* = 8 rats/group. *P < 0.05.

**Figure 4:** LPS causes upregulation of PRDX1* in vitro.* (a) Morphological changes in BEAS-2B cells after treatment with 1 *μ*g/mL or 10 *μ*g/mL LPS in 12 hours or 24 hours. BEAS-2B without any treatment was used as a control, original magnification, ×200. (b) Effects of LPS on cell viability. Results are presented as the percentage absorbance of the control group. Data are expressed as the means ± SD. *P < 0.05 versus the control group. (c) and (d) the expression of PRDX1 in culture media was evaluated by western blotting (c) and ELISA (d) after challenge with LPS. *α*-Tubulin was not detected in the conditioned media. Experiments in (c) and (d) were repeated at least 3 times, with similar results. Each bar represents the mean ± SD of three independent experiments.*P < 0.05.

**Figure 5:** PRDX1 expression modulated inflammation in airway epithelium cells. (a) Overexpression of PRDX1 in BEAS-2B cells was analyzed by WB. *β*-Actin was used as a loading control. (b) Knockdown of PRDX1 in BEAS-2B cells was analyzed by WB. *β*-Actin was used as a loading control. Mock: cells were transfected with transfection reagent alone; shRNA-NC: cells were transfected with a shRNA vector. (c) Overexpression of PRDX1 increased the expression of proinflammatory cytokines. RT-PCR analysis of expression of IL-6, IL-8, and TNF-*α* in vector or pMSCV-PRDX1 transduced BEAS-2B cells treated with LPS or control. (d) Knockdown of PRDX1 inhibited the expression of proinflammatory cytokines. RT-PCR analysis of expression of IL-6, IL-8, and TNF-*α* in pSUPER-shRNA NC or pSUPER-shPRDX1#3 treated with LPS or control. (e) Expression of p65 in nuclear extracts of indicated cells was analyzed by western blotting. p85 was used as a loading control. Experiments were repeated at least 3 times, with similar results. Each bar represents the mean ± SD of three independent experiments.*P < 0.05.

**Table 1:** Primer sequences used reverse transcription-PCR.

primers	sequences
GAPDH forward	5′-TCCTCCACCTTTGACGCT-3′
GAPDH reverse	5′-TCTTCCTCTTGTGCTCTTGC-3′
Peroxiredoxin1 forward	5′-GGAGGATTGGGACCCATGAAC-3′
Peroxiredoxin1 reverse	5′-AGAGCGGCCAACAGGAAGATC-3′
IL-6 forward	5′-GGAGACTTGCCTGGTGAA-3′
IL-6 reverse	5′-CTGAGGTGCCCATGCTAC-3′
IL-8 forward	5′-TGGCAGCCTTCCTGATTT-3′
IL-8 reverse	5′-CTTCTCCACAACCCTCTG-3′
TNF-*α* forward	5′-CGAGTCTGGGCAGGTCTA-3′
TNF-*α* reverse	5′-AGCCGTGGGTCAGTATGTGAGA-3′

**Table 2:** The classification of differential proteins in ALI lung tissue with the comparison of control group.

Protein name	Accession number	Protein MW (Da)	Regulation	Fold change
(A) Metabolism protein				
Glyceraldehyde-3-phosphate dehydrogenase	gi|8393418	35805.2	Up	2.13
Phosphoglycerate kinase 1	gi|40254752	44510	Up	2.32
Aldehyde dehydrogenase, mitochondrial	gi|45737866	55566.2	Up	2.07
Nucleoside diphosphate kinase B	gi|55926145	17271.9	Up	2.03
Malate dehydrogenase	gi|37590235	36461	Down	2.31
Aldolase A	gi|202837	39235.3	Up	2.20
(B) Antioxidant				
Superoxide dismutase2	gi|8394331	24658.6	Up	2.57
Peroxiredoxin 1	gi|16923958	22095.3	Up	4.79
Glutathione S-transferase alpha-4	gi|157820217	25493.4	Down	2.88
(C) Binding proteins				
Lectin, galactose binding, soluble 5	gi|6981154	16186	Down	2.86
Transthyretin	gi|20663827	13589.8	Down	2.70
Apolipoprotein E	gi|37805241	35741.4	Down	2.44
Calreticulin	gi|253851	29142.4	Up	2.40
Selenium-binding protein 1	gi|18266692	52498.4	Down	2.73
Vitamin-D binding protein	gi|203941	53482	Up	2.77
Haptoglobin	gi|60097941	38538.5	Up	3.1
(D) Signal transduction				
Rho-associated protein kinase 1	gi|13592049	159526.6	Down	2.72
Translationally controlled tumor protein	gi|6678437	19449.6	Up	2.94
